# The Association of Vitamin D Status with Dyslipidaemia and Biomarkers of Endothelial Cell Activation in Older Australians

**DOI:** 10.3390/nu8080457

**Published:** 2016-07-28

**Authors:** Ali M. Alyami, Virginie Lam, Mario J. Soares, Yun Zhao, Jillian L. Sherriff, John C. Mamo, Anthony P. James, Fiona Coombes

**Affiliations:** 1 Health Promotion & Disease Prevention, School of Public Health, Curtin Health Innovation Research Institute, Faculty of Health Sciences, Curtin University, Perth 6102, Australia; alimahdim.alyami@postgrad.curtin.edu.au (A.M.A.); virginie.lam@postgrad.curtin.edu.au (V.L.); J.Sherriff@curtin.edu.au (J.L.S.); J.Mamo@curtin.edu.au (J.C.M.); T.P.James@curtin.edu.au (A.P.J.); 2 Occupation and the Environnent, School of Public Health, Faculty of Health Sciences, Curtin University, Perth 6102, Australia; Y.Zhao@exchange.curtin.edu.au; 3 University Health Service, Support Services, Curtin University, Perth 6102, Australia; F.Coombes@exchange.curtin.edu.au

**Keywords:** vitamin D, endothelial function, inflammation, cardiovascular disease, lipids

## Abstract

Background/Aims: Vitamin D has been investigated for many non-skeletal effects. The objective of this study was to determine whether circulating lipids, systemic inflammation, and biomarkers of endothelial cell activation varied with the vitamin D status of older Australians. Methods: One hundred and one participants were proportionately and randomly sampled across tertiles of 25 hydroxy vitamin D (25(OH)D) from a larger cohort of free living older adults (T1 median = 97; T2 median = 74.5; T3 median = 56.8 nmol/L). Overnight fasting blood samples were assayed for 25(OH)D, parathyroid hormone (PTH), insulin, triacylglycerol (TAG), total cholesterol (TC), low density lipoprotein cholesterol (LDL-C) and high density lipoprotein cholesterol (HDL-C). Markers of systemic inflammation (high sensitivity C-reactive protein (hsCRP), tumour necrosis factor-α (TNF-α)) and endothelial activation (hepatocyte growth factor (HGF), P-selectin and soluble vascular cell adhesion molecule (sVCAM), soluble intracellular adhesion molecule (sICAM)) were determined. A general linear model multivariate analysis with a backward elimination procedure was performed. Results: Eighty-three participants (48 women, 35 men), aged 65 ± 7.7 years, BMI 28 ± 4.5 kg/m^2^, with complete data were analyzed. The final parsimonious model controlled for age, gender, BMI, and McAuley’s index, but excluded season, medications, and PTH. There were significant differences across 25(OH)D tertiles in TC (T1 < T3, *p* = 0.003; T2 < T3, *p* = 0.001), LDL-C (T1 < T3, *p* = 0.005; T2 < T3, *p* = 0.001), TAG (T2 < T3, *p* = 0.026), HGF (T1 > T3, *p* = 0.009) and sVCAM (T1 > T3, *P* = 0.04). Conclusions: Higher vitamin D status may protect the endothelium through reduced dyslipidaemia and increased HGF.

## 1. Introduction

The 2011–2012 National Health Survey [1] revealed that most Australian adults were vitamin D sufficient, as judged by levels of 25 hydroxy vitamin D (25(OH)D) > 50 nmol/L, with only 23% having inadequate status. However, older Australians had a higher prevalence of inadequacy [1,2]. Contributing factors include limited sun exposure due to an increased awareness of skin cancer; skin pigmentation; genetic determinants; adiposity, illness, or immobility resulting in indoor living; age-related decline in the skin’s ability to synthesize vitamin D; and dress habits [3,4].

The recommended level of 25(OH)D that signals vitamin D sufficiency is based on a value required for bone health [5], however there is growing interest in recommendations that optimize extra-skeletal outcomes, including cardiovascular health. The precise mechanism(s) whereby vitamin D status may modify the development of atherosclerosis are unknown [6], however there is evidence for roles in both endothelial function and plasma cholesterol levels [6]. The impact of vitamin D status on LDL-cholesterol (LDL-C) and total cholesterol (TC) remains equivocal due to the randomized controlled trials (RCT) published to date having small numbers of subjects, variable doses of vitamin D, a wide-range of intervention times, and a relative lack of participants with low vitamin D status at baseline [7].

The impact of inflammation on endothelial function is well recognized [8] and the understanding of the immune system’s metabolism of vitamin D has exploded over the last five years [9]. Unlike many other cell types in the body, various immune cells can hydroxylate 25(OH)D, with the availability of 25(OH)D regulating the synthesis of the active form, 1,25 di-hydroxy vitamin D (1,25(OH)_2_D or calcitriol) rather than the hormonal regulation that characterizes renal synthesis [9]. Furthermore, unlike renal synthesis, there is a lack of negative feedback resulting in locally elevated levels of 1,25(OH)_2_D [9]. Immune cells express vitamin D receptors (VDR) and can therefore respond to 1,25(OH)_2_D, although T cells need to be activated before the VDR gene is expressed [10]. In a similar manner, the endothelium expresses VDR and has the enzymatic machinery to locally produce the active hormone 1,25(OH)_2_D from circulating 25(OH)D. Hence the endothelium also does not have a feedback control system, and synthesis of the hormone depends on the level of circulating 25(OH)D [6].

There are many systemic inflammation biomarkers and endothelial cell activation molecules that have been studied as surrogates for cardiovascular disease risk [11]. Commonly measured markers include tumour necrosis factor-alpha (TNF-α), high sensitivity C-reactive protein (hsCRP), leptin, soluble intracellular adhesion molecule (sICAM-1) and soluble vascular cell adhesion molecule (sVCAM-1), hepatocyte growth factor (HGF), and selectins (P and E-selectin), all of which are increased with the inflammatory state [12,13]. In general, higher levels of these biomarkers are considered to be independent risk factors for cardiovascular disease (CVD) [14], and vitamin D deficiency may lead to elevated levels of these biomarkers [13,15]. We and others have recently reviewed the data in the area and concluded that there is limited causative evidence to link 25(OH)D levels to systematic inflammation and endothelial dysfunction [6,13]. The purpose of this study is to investigate the potential links between dyslipidaemia, endothelial cell activation, and vitamin D status in older Australians.

## 2. Experimental Section

### 2.1. Subject Selection

One hundred and one participants were proportionately and randomly sampled across tertiles (T1 = highest, T2 = middle, T3 = lowest) of 25(OH)D from a larger cohort of free living older adults [16]. These participants were of European origin and residents of Perth, Western Australia. The primary study had ethical approval from the Curtin University Human Ethics Committee (approval number HR97/2011), and all participants provided informed written consent. The study was conducted between December 2011 and August 2012, a period that coincided with one of the hottest years in Perth.

### 2.2. Blood Analysis

Overnight fasted venous blood was collected at PathWest, Royal Perth Hospital for measurement of insulin, triacylglycerol (TAG), total cholesterol, and lipid fractions. Serum 25(OH)D was measured with a kit from Immunodiagnostic Systems, Boldon, UK. The kit quantifies all hydroxylated forms of vitamin D. The 25(OH)D kit had a sensitivity of 5 nmol/L with an intra-assay CV of 5.3%–6.7% and inter-assay CV of 4.6%–8.7%. Parathyroid hormone (PTH) was measured using a kit from Immutopics Inc., San Clemente, CA, USA. The PTH kit had a detection limit of 13 pg/mL, with intra-assay CV of 3%–5% and inter-assay CV of 4.7%–7.4%.

Markers of systemic inflammation and endothelial activation, e.g., hsCRP, TNF-α, HGF, P-selectin, sVCAM, sICAM, and leptin, were measured at the School of Public Health, Curtin University using a Human Adipokine Magnetic Bead Panel 2 (HADK2MAG-61K) and Human Cardiovascular Disease Magnetic Bead Panel 2 (HCVD2MAG-67K) and were run on a MAGPIX system (Merck Millipore, Luminex, Austin, TX, USA). Intra-assay CVs ranged from 3% for TNF-α to 5% for leptin, and inter-assay CVs ranged from 11% for insulin to 19% for TNF-α.

### 2.3. Statistical Analysis

The main outcome variables of this study were total cholesterol (TC), LDL-cholesterol, high density lipoprotein (HDL)-cholesterol, TAG, D-Dimer, sICAM, MPO, P-selectin, sVCAM, leptin, TNF, CRP, and HGF. The primary variable of interest was 25(OH)D, which was categorized into tertiles (T1 = highest, T2 = middle, T3 = lowest). Normality was assessed for all outcome variables and natural logarithm (or square root) transformation was applied if severe skewness was observed. One-way ANOVA was used to compare the differences between the tertiles for characteristics of subjects. Multivariate ANCOVA (MANCOVA) involved in multivariate general linear model (GLM) was used to test for differences in the main outcomes between tertiles of 25(OH)D, controlling initially for age, gender, BMI, McAuley’s index, season, medications, and PTH. In the regression modelling, a backward elimination approach was then applied and variables that did not contribute to the model were removed at a 5% significance level. The final parsimonious model retained age, gender, BMI, and McAuley’s index as significant confounders. Where overall significant effects were obtained, individual category comparisons were carried out separately for T1 and T2 against the lowest vitamin D tertile (T3), as a reference. McAuley’s index and QUICKI were strongly related in our sample (*r* = 0.843; *p* = 0.001). We preferred McAuley’s index since it was more strongly related to lipid endpoints in this study as compared to QUICKI (data not shown). Importantly, other authors have also endorsed its usefulness in reflecting aspects of insulin sensitivity in different population groups when compared to the gold standard clamp technique [17,18,19]. All analyses were performed using IBM SPSS Statistics for Windows, Version 22.0 (IBM Corp. Released 2013, Armonk, NY, USA) [20]. A significant difference was inferred when *p* values were less than 0.05.

## 3. Results

Eighty-three participants with complete data entered the final analysis. General characteristics of these volunteers are provided in Table 1.

### 3.1. 25(OH)D and Lipids Profiles

Based on the multivariate regression model, significant differences were found across 25(OH)D tertiles in TC (T1 < T3, *p* = 0.003; T2 < T3, *p* = 0.001) and LDL-C (T1 < T3, *p* = 0.005; T2 < T3, *p* = 0.001). HDL-C was not significantly different amongst the tertiles (Table 2). While a difference in TAG (T2 < T3, *p* = 0.04) was noted, the MANOVA only showed an overall trend (*p* = 0.082) for the effect of 25(OH)D on TAG (Table 2).

### 3.2. Systemic Inflammatory Biomarkers and Endothelial Cells Activation Molecules

The multivariate regression model also revealed significant differences across 25(OH)D tertiles in HGF with T1 > T3 (*p* = 0.009, Table 3). While MANOVA showed that sVCAM in T1 is greater than that in T3 on average (T1 > T3 *p* = 0.04), the overall MANOVA effect of 25(OH)D on sVCAM only approached significance with a *p* value of 0.091 (Table 3). There were no other significant differences detected. Further adjustment for TNF-α and/or hsCRP did not modify any of these outcomes (data not shown).

## 4. Discussion

Cardiovascular disease (CVD) is a significant contributor to the adverse health profile of Western Australians [21] and accounts for much of the State’s health expenditure. Besides traditional serum lipid profiles and systemic inflammatory markers, endothelial dysfunction may underscore CVD, and measurement of endothelial cell activation could be important in determining this risk. A working model would hence place elevated TNF-α and hsCRP as indicators of systemic inflammation, and the pro-atherogenic state that occurs with dyslipidaemia would engender endothelial cell dysfunction and increased endothelial cell activation [22]. The latter would manifest as increased circulating levels of a variety of markers, including soluble vascular adhesion molecules, the selectins, pro-atherogenic D-dimer and myeloperoxidase (MPO). Adequate 25(OH)D would then offset systemic inflammation, while potentially returning the endothelium to its quiescent state [6].

The majority of our older participants had a sufficient vitamin D status (25(OH)D > 50 nmol/L) as judged by current criteria [23,24]. This was not due to vitamin D supplement use, but could reflect the higher than normal annual temperature that year in Perth, where average annual temperatures of 25–26 °C were common on the coastal plain. We observed that higher tertiles of 25(OH)D were found to be associated with lower TC and LDL-C. Such data would argue that 25(OH)D is potentially protective of CVD risk even when vitamin D status is well above the recommended level (Table 2). There are now several studies that have examined the effect of vitamin D on lipid endpoints. Cross-sectional studies have indicated inverse associations between 25(OH)D and TAG [25] and a direct positive relationship with HDL-C [26]. Zimmerman et al. (2011) systematically reviewed the literature and concluded that cross-sectional studies favored the finding of a lower TAG, especially in studies where participants started from a higher TAG concentration [27]. Similarly, based on a very large dataset from one laboratory, Lupton et al. (2015) observed a significant inverse relationship between higher 25(OH)D and all circulating lipid markers [28]. The results of a meta-analysis of RCTs only partially confirmed these observational outcomes. While Chaloumas et al. (2014) found no impact of vitamin D supplementation on lipid markers [29], Manousopoulou et al. (2015) found a significant decrease in TAG [30]. In contrast, the latter review also reported a small increase in LDL-C with vitamin D [30]. Clearly, RCTs do not support a beneficial effect, while reviews of cross-sectional studies all show a decrease in TAG in particular. Hence, while our results are suggestive of a beneficial effect, a causal link between these observations requires further study for clarification [31].

Vitamin D could have a beneficial effect on endothelial function through a variety of effects including lowering systemic inflammation through reductions in TNF-α and hsCRP [32,33,34,35], and in decreasing endothelial cell activation as judged by lower sICAM-1 and sVCAM-1 [34,35]. Vitamin D may also increase plasma leptin, which could be vasodilatory to the endothelium [36,37]. Furthermore, low 25(OH)D levels leads to dysregulation in neutrophil activity leading to increased MPO levels [38]. On the other hand, 25(OH)D shows no correlation with P-selectin levels in the blood [32,34]. Endothelial cell activation molecules are indications of arterial health and function. These molecules—D-dimer, sICAM-1, sVCAM-1, MPO, P-selectin, and HGF—are amongst a host of others that have been used to study endothelial cell functioning [6,11,13]. While each molecule has a different role in the endothelium, in general they all show an increase with endothelial inflammation [39,40,41,42,43,44,45,46,47]. Contrary to our hypothesis, we found little significant evidence to support an association of 25(OH)D with most markers of endothelial cell activation that were measured (Table 3). In fact, with one marker, we observed a trend for the reverse; that those in the highest tertile of 25(OH)D had significantly higher sVCAM relative to the reference group (Table 3). However, it must be noted that the overall effect was marginally significant (Table 3). These outcomes did not change with further adjustment for inflammatory markers, TNF-α or hsCRP.

sVCAM-1 is expected to reflect membrane bound VCAM, which is involved in leukocyte migration, an early step in atherosclerosis. Although non-significant, the data may reflect the potential deleterious effects of very high levels of 25(OH)D. Interestingly, we also found that at these circulating levels of 25(OH)D (Tertile 3), HGF increased significantly more than in the reference group (Table 3). HGF has a major role in the endothelium, and is a potent angiogenic factor. It has the added benefit of preventing increased vascular permeability and leukocyte adhesion that is observed with another growth factor, vascular endothelial growth factor (VGEF). In fact, combination therapy of VGEF and HGF has been proposed for CVD [48]. It is possible that the increase in HGF at the highest tertile is a compensatory/adaptive response to counter deleterious effects of sVCAM.

## 5. Limitations

The cross-sectional nature of the study limits generalization and does not offer causation. Since this population group had relatively good vitamin D status and our sample was relatively small, we were constrained in detecting potential differences in those with very poor vitamin status. Furthermore, as measures of habitual physical activity were unavailable, we could not control for its effect on CVD risk markers. As a fat-soluble vitamin, the potential deleterious effects of too high a status may also need consideration. While there is some evidence that 25(OH)D status and CVD mortality may be represented by a non-linear, reverse J shaped association [49], emerging long term data do not support this view [50].

## 6. Conclusions & Future Directions

Higher vitamin D status was associated with lower circulating lipid levels, namely lower total and LDL-cholesterol, and potentially lower TAG. In contrast, a higher circulating HGF may have a protective role in the endothelium. Future randomized controlled trials on a larger sample of patients with initial low vitamin D status would confirm whether vitamin D has a causal relationship with endothelial dysfunction. In this regard, a recent 4-month RCT on those at risk of type 2 diabetes found a significant improvement in arterial stiffness following both vitamin D_2_ and vitamin D_3_ supplementation [51]. Such data emphasize the potential impact of the long term outcomes of the VITAL trial [52].

## Figures and Tables

**Table 1:** General characteristics of the study participants across tertiles of vitamin D status.

Variable	Tertile 1 (*N* = 25)	Tertile 2 (*N* = 29)	Tertile 3 (*N* = 29)	*p* Value
25(OH)D (nmol/L)	97.00 (83.00–202.60)	74.50 (66.00–83.00)	56.8 (26.34–65.42)	
Age (years)	65.85 (1.44)	65.12 (1.44)	64.96 (1.44)	0.720
Gender (M/F)	13 (39.4)/20(60.6)	11 (33.3)/22 (66.7)	20 (57.1)/15 (42.9)	0.119
Weight (kg)	81.38 (2.60)	78.27 (2.42)	76.34 (2.42)	0.945
BMI (kg/m^2^)	28.18 (0.91)	28.45 (0.84)	27.62 (0.84)	0.609
SBP (mmHg)	148.12 (4.26)	143.00 (3.95)	142.69 (3.95)	0.734
DBP (mmHg)	84.52 (2.07)	80.14 (1.93)	81.41 (1.93)	0.387
PTH (pmol/L)	7.7 (13.88)	4.7 (2.74)	6.2 (4.81)	0.421
McAuley’s index	8.3 (2.21)	8.3 (2.26)	8.3 (2.17)	0.999

Data are mean (SD) if continuous, except 25(OH)D [25 hydroxy vitamin D] which is median (range). BMI, body mass index; SBP, systolic blood pressure; DBP, diastolic blood pressure; PTH, parathyroid hormone.

**Table 2:** Vitamin D status and lipids profiles in older Australians.

Marker	Tertile 1 (*N* = 25)	Tertile 2 (*N* = 29)	Tertile 3 (*N* = 29)
25(OH)D (nmol/L)	97.0 (83.00–202.6)	74.5 (66.00–83.0)	56.8 (26.34–65.42)
TC (mmol/L)	4.87 ** (4.18–5.83)	4.91 † (3.92–5.85)	5.91 (4.52–6.48)
LDL-C (mmol/L)	2.80 ** (2.31–3.69)	2.79 † (2.16–3.55)	3.64 (2.60–4.09)
TAG (mmol/L) ^1^	1.16 (0.46–2.60)	1.13 * (0.40–2.57)	1.37 (0.52 –2.50)
HDL-C (mmol/L)	1.30 (0.98–1.86)	1.43 (1.05–1.82)	1.45 (1.09–1.86)

Data are predicted median (range) from MANCOVA model that initially adjusted for age, gender, BMI, McAuley’s index, season, medications, and PTH, but season, medications, and PTH were excluded in the final model by a backward elimination procedure. ^1^ Overall MANOVA, *p* = 0.082 for triacylglycerol (TAG), but *p* < 0.05 for total cholesterol (TC) and low density lipoprotein cholesterol (LDL-C). High density lipoprotein cholesterol (HDL-C) was non-significant. Post-hoc tests * *p* < 0.05; ** *p* < 0.005; † *p* < 0.001; vs. Tertile 3.

**Table 3:** Systemic inflammatory and endothelial biomarkers across tertiles of vitamin D status.

Marker	Tertile 1 (*N* = 25)	Tertile 2 (*N* = 29)	Tertile 3 (*N* = 29)
25(OH)D (nmol/L)	97.0 (83.0–202.6)	74.5 (66.0–83.0)	56.8 (26.3–65.4)
TNF–α (pg/mL)	5.40 (3.80–9.12)	4.40 (3.10–6.00)	4.10 (3.10–6.46)
CRP (ng/L)	2134.50 (933.00–9120.00)	2079.00 (891.00–4467.00)	2359.00 (1122.0–9550.0)
Leptin (pg/mL)	7952 (4074–79433)	11871.4 (3020–40738)	8323.40 (2692–51286)
D–dimer (pg/mL)	2538 (1318–3162)	2258 (1513–3548)	1958 (1122–3630)
sICAM-1 (pg/mL)	126.00 (109.6–144.5)	114.40 (95.5–141)	132.77 (117.5–158.5)
MPO (pg/mL)	358.00 (302.00–447.00)	309.00 (219.00–417.00)	399.00 (288.40–489.80)
P-selectin (pg/mL)	130.00 (115.00–186.00)	141.00 (100.00–199.50)	159.00 (104.70–195.00)
sVCAM-1 (pg/mL) ^1^	877.00 * (708.0–955.00)	705.80 (616.50–832.00)	703.00 (602.60–891.30)
HGF (pg/mL)	512.50 ** (355.00–633.50)	351.60 (263.00–509.00)	318.50 (219.00–426.80)

Data are predicted median (range) from MANCOVA model that initially adjusted for age, gender, BMI, McAuley’s index, season, medications and PTH, but season, medications and PTH were excluded in the final model by a backward elimination procedure. ^1^ Overall MANOVA, *p* = 0.091 for sVCAM but *p* < 0.05 for HGF. Post-hoc tests * *p* < 0.05; ** *p* < 0.01 vs. Tertile 3. TNF-α, tumor necrosis factor-alpha; CRP, C reactive protein; sICAM, soluble intracellular adhesion molecule; MPO, myeloperoxidase; sVCAM, soluble vascular cell adhesion molecule; HGF, hepatocyte growth factor.
